# EEG biofeedback improves attentional bias in high trait anxiety individuals

**DOI:** 10.1186/1471-2202-14-115

**Published:** 2013-10-07

**Authors:** Sheng Wang, Yan Zhao, Sijuan Chen, Guiping Lin, Peng Sun, Tinghuai Wang

**Affiliations:** 1 Department of Physiology, Zhongshan School of Medicine, Sun Yat-sen University, Guangzhou, People’s Republic of China

**Keywords:** EEG Biofeedback, Anxiety, Event-related potentials, P300, Attention

## Abstract

**Background:**

Emotion-related attentional bias is implicated in the aetiology and maintenance of anxiety disorders. Electroencephalogram (EEG) biofeedback can obviously improve the anxiety disorders and reduce stress level, and can also enhance attention performance in healthy subjects. The present study examined the effects and mechanisms of EEG biofeedback training on the attentional bias of high trait anxiety (HTA) individuals toward negative stimuli.

**Results:**

Event-related potentials were recorded while HTA (n=24) and nonanxious (n=21) individuals performed the color-word emotional Stroop task. During the emotional Stroop task, HTA participants showed longer reaction times and P300 latencies induced by negative words, compared to nonanxious participants.

The EEG biofeedback significantly decreased the trait anxiety inventory score and reaction time in naming the color of negative words in the HTA group. P300 latencies evoked by negative stimuli in the EEG biofeedback group were significantly reduced after the alpha training, while no significant changes were observed in the sham biofeedback group after the intervention.

**Conclusion:**

The prolonged P300 latency is associated with attentional bias to negative stimuli in the HTA group. EEG biofeedback training demonstrated a significant improvement of negative emotional attentional bias in HTA individuals, which may be due to the normalization of P300 latency.

## Background

Trait anxiety is characteristic of personalities associated with a tendency to experience anxiety. Excessive trait anxiety is a risk factor for anxiety disorder and other psychosomatic diseases [1,2]. Many behavioral studies have demonstrated that negative emotional stimuli interfere with attention performance in anxious individuals [3-5]. The color-word emotional Stroop task is an effective experimental method of assessing interference between emotion and attention [6,7]. A number of studies have shown that anxious individuals respond more slowly to negative words than do healthy controls, suggesting that anxious individuals tend to allocate their attention selectively toward negative-related information [5,8]. This attentional bias may play an important role in the onset and maintenance of anxiety disorders. However, an effective way to control or improve this emotion-related attentional bias in high trait anxiety (HTA) individuals is still undetermined.

Electroencephalogram (EEG) biofeedback refers to an operant conditioning paradigm that participants learn in order to alter their brain activity by regulating specific parameters of the EEG; this process is intended to improve neurological and psychiatric symptoms. Several studies have demonstrated the clinical value of EEG biofeedback in treating psychological disorders such as anxiety [9,10], epilepsy [11] and attention deficit hyperactivity disorder [12], as well as optimising the psychoemotional status and cognitive performance of healthy subjects [13,14]. Predominant alpha (8–13 Hz) amplitude occurs in a relaxed and eye-closed state, moreover, it is related to the idling of the brain while remaining ready for engagement [15]. The decrease in alpha amplitude observed in opened eyes indicates an increase in activation, whereas the increase in alpha amplitude in closed eyes indicates less activation [16]. Amplitude of the alpha band reflects an inhibition of irrelevant information which in turn may facilitate performance on the task [17]. Eye-closed neurofeedback training aimed at increasing alpha amplitude/power may lead to selective inhibition of irrelevant attentional activity and an improvement of neural efficiency [15]. An increase in alpha power is the most commonly used indicator of relaxation as a means to reduce anxiety [10,18,19] and enhance short term memory performance [20]. However, the effectiveness of EEG biofeedback using alpha training directed toward the attentional bias in anxious individuals remains unknown.

The assessment of attention performance and EEG activity using alpha training may be of great value in providing an empirical rationale for clinical application of EEG biofeedback to specific symptoms. Egner and Gruzelier [21] showed that EEG biofeedback training led to significant changes in attention performance and event-related potentials (ERPs) in healthy volunteers. Beta protocol learning was positively correlated with increased target P300 ERPs in an auditory oddball task. P300 ERPs are thought to reflect the attentional and mental state in task execution process of information collection and classification (eg. working memory and cognitive function, respectively) [22]. Recent finding indicated that the P300 in the target condition was modulated by the changes of alpha event-related desynchronization, involving attention allocation [23]. Furthermore, alpha band activity is strongly related to P300, which suggests that the P300 is related to attention and memory processing. The P300 may result from the operation of neural inhibition generated when cognitive mechanisms are engaged by stimulus and task demands [24], but the relation between P300 and attentional bias in HTA individuals is still unclear. It is also unknown whether changes in alpha activity and associated P300 of HTA individuals may in some way mediate their attentional bias.

To investigate the efficacy and mechanisms of EEG biofeedback training on attentional bias of HTA individuals to negative stimuli, the present study will apply EEG biofeedback using alpha training to HTA individuals and examine its effect on attentional bias associated with brain activity. In addition, we assessed the specific change of P300 latency during the emotional Stroop task after EEG biofeedback.

## Methods

Participants were recruited from a pool of 358 undergraduates at Sun Yat-Sen University, who were administered with the Chinese version of the State-Trait Anxiety Inventory (S-TAI, Spielberger et al., 1983). According to the TAI’s score, participants were classified into the HTA group with 20% of the highest scores (N=24, 14 females) and the nonanxious (NA) group with 20% of the lowest scores (N=21, 11 females). All participants were right-handed as determined by the Annett Handedness Inventory (Annett M., 1976). They were all native Chinese speakers with self-reported normal color vision. Participants were informed of the procedures of the study and gave written informed consent. They declared no previous personal history of neurological and psychiatric disorder or of familial psychiatric disorder. This study was approved by the Ethics Committee of the Sun Yat-Sen University.

### Emotional Stroop task (EST)

Word presentation and response recording were controlled by E-Prime software (Psychological Software Tools, Pittsburgh, PA). The experimental materials consisted of positive, negative and neutral words presented in different colors (red, green and blue). There were 30 trials for each color (red, green and blue) and valence (negative, positive and neutral) category; thus there were 270 trials in total. The emotional and neutral words were selected from the Chinese Affective Word System [25]. Each condition comprised 15 words; three word types were matched for arousal, word frequency and complexity of the characters. The size of the Chinese words was Song Ti No.20. Each trial consisted of one word presented in the center of a 19-inch screen on a black background in a pseudo-random order.

Participants were seated in a dark room facing a monitor placed 60 cm from their eyes. They were instructed to rest their fingers on the “F”, “J” and Space buttons on the keyboard; each of the three buttons was respectively designated to indicate red, green or blue color. These stimulus–response key assignments were counterbalanced across individuals. All participants were told that a white cross would appear in the center of the screen serving as a fixation point, followed by one word written in color. The fixation point lasted for 300–500 ms and then each word for 1500 ms. Participants were asked to ignore the meaning of the words and identify the color as quickly as possible by pressing the designated button of the corresponding color. The experiment was divided into a practice phase and a test phase. The practice phase was designed to rehearse the mapping of colors onto fingers and pressing of the response buttons. When the accuracy rate for each individual reached 85%, the practice phase was ended. The formal test phase consisted of three blocks. Each block had 90 judgment trials presented in individually varied, randomized sequences. Participants were instructed to try their best to avoid blinking or any eye movement and keep their eyes fixated on the monitor rather than look down at their fingers during trial phases. After each block, there was a period of brief rest.

### ERP recording and analysis

EEG data were recorded from 64 scalp sites with an ERP workstation (Brain Products) using tin electrodes mounted in an elastic cap during the EST. Electrodes were referenced to linked earlobes (off-line) and the ground electrode was placed 1.5 cm anterior to the central frontal (Fz) electrode. Impedance was kept below 5 kΩ. Data were digitized at a sampling rate of 500 Hz and passed through a 0.05-80 Hz bandpass filter. Recording, digitization and subsequent off-line data processing were carried out with Brain Vision System (Version 1.05 Software, Brain Products GmbH, Germany).

Corrected data were divided into periods of 900 ms, starting with 100 ms prior to the stimulus onset. Epochs were baseline corrected with the 100 ms pre-stimulus interval, and any epochs containing EEG fluctuation exceeding ±80 μV were rejected as artifact contamination. Only trials of correct responses were used in the analysis. A minimum of 40 trials was available for each condition. On the basis of the ERPs grand averaged waveforms and a topographic map, the following nine electrode sites were chosen for statistical analysis: C3, Cz, C4, P3, Pz, P4, O1, Oz and O2. The P300 wave was defined as the highest positive deflection at the central, parietal and occipital electrodes within a post-stimulus time interval of 250–400 ms for attended target stimuli.

### Experiment 1

The between-subject independent variable was the group (HTA and NA), within-subject independent variable was the word type (negative, positive and neutral). The dependent variable was the reaction time or P300 latency in naming the color words in the EST. We quantified attentional bias as reaction time in naming the color words during the EST. The working hypothesis was that if there were any attentional bias induced by the emotional words as a cue, the reaction time would be increased or decreased. The ERP waves from the three word types were overlapped and averaged separately, and then P300 latencies were compared between the HTA and NA groups.

### Experiment 2

The HTA individuals in experiment 1 were randomly divided into two groups, EEG biofeedback (EEG BF) group (n=12) for 8–13 Hz alpha training, and sham biofeedback (sham-BF) group (n=11), without EEG feedback. Both groups received the same duration and frequency of the protocols for twice a week and a total of 15 times. The two groups completed the S-TAI measurement and the EST during ERP recording after the intervention. Pre- and post- training ERP recordings were carried out at approximately the same time of day for the HTA individuals and inter-test intervals exceeded 12 weeks. A Group (EEG BF and Sham-BF)×Word type (negative, positive and neutral)×Time (pre- and post-intervention) mixed-design analysis of variance (ANOVA) was applied, followed by post hoc comparisons assessing within-group changes for each group (paired t-tests), and between-group differences (independent t-tests).

### EEG biofeedback

EEG biofeedback training was conducted with a spirit Nexus-16B (Netherlands Spirit-Ming) and its software (Biotrace+ version 1.20, Mind media B.V. Netherlands). A signal was acquired at 160 Hz, A/D converted and band-filtered to beta (14–18 Hz), alpha (8–13 Hz) and theta (4–7 Hz) components. According to the international 10–20 system, the active scalp electrode was placed at C3 or C4 for alpha training with a reference electrode placed ipsilaterally and a ground electrode placed on the contralateral earlobe. Impedance was kept below 5 kΩ. A 3-5min eye-closed baseline was first recorded during pre-feedback to set initial alpha band thresholds. Subsequently, eye-closed auditory feedback was engaged for 27 min continuously. Alpha activity was represented by an ‘ocean waves’ background sound and over-threshold alpha activity by a ‘warble’ sound; the latter was set to have a higher priority over the former. Over-threshold alpha-related sounds acted as a reward and were intended for relaxation. The more alpha activity exceeded threshold, the greater the feedback sound. The reward band threshold was set within a range of 0.7 to 1.5 times its baseline average. This range ensured that the participants would not be rewarded for simply tensing cranial muscles. Artifact rejection thresholds were set for each individual and auditory feedback signals were not heard within 5 seconds of eye movements or other motor activity, as they would have caused gross EEG fluctuations.

The working principles of the feedback loop were explained to the participants in the EEG BF group. Subjects wore a set of headphones and rested in a comfortable reclining chair. They were instructed to relax deeply to achieve an increase in the amount of alpha band activity resulting from sound representation, but to prevent the subject from falling asleep. EEG inhibition of delta band (1–4 Hz) activity was also implemented to preclude the latter. The sham-BF participants were provided with only the ‘ocean waves’ background sound during the whole training. All subjects participated in twice-weekly training sessions over the course of 8 weeks.

## Results

### Experiment 1

#### Baseline data

There were no statistically significant differences between the HTA and NA groups for gender, age or educational level (*p* >0.05). Total scores of the S-TAI were significantly higher in the HTA group than in the NA group (Table 1).

**Table 1:** Comparison of baseline data between the HTA and NA groups

**Item**	**HTA Mean±SD**	**NA Mean±SD**	***X***^**2**^	**t**	***p***
Gender (male/female)	10 / 14	10 / 11	0.02		0.90
Age (y)	20.38±0.88	20.43±0.87		−0.21	0.84
Educational level (y)	14.08±0.28	14.10±0.30		−0.14	0.89
TAI score	57.04±3.95	32.48±2.25		25.13	0.00
SAI score	52.50±8.42	32.38±4.43		9.82	0.00

#### Behavioral data

The accuracy rates for naming the color words were above 90% in both groups. Reaction time (RT) for negative, positive and neutral word trials was analyzed for correct trial responses between 300 and 1200 ms. A Word type (negative, positive, neutral)×Group (HTA and NA) repeated measure ANOVA was conducted. RTs were the dependent variable. Greenhouse–Geisser corrections were inspected. There was a significant main effect of word type on RTs (F(2, 70)=5.56, *p*=0.006). The interaction between word type and group was significant (F(2, 70)=3.45, *p*=0.037), indicating that the group difference of attentional effect was dependent on emotional stimuli. Simple-effect tests revealed that RTs toward negative words were longer in the HTA group compared to the NA group (F(1, 35)=5.09, *p*=0.03). Moreover, RTs for negative words were longer than for neutral words in the HTA group (F(1, 35)=4.12, *p*=0.04) (Figure 1), but there was no significant effect in the NA group.

**Figure 1:** **Comparison of reaction time (RT) in the EST between the HTA and NA groups.** The RT for negative words was longer in the HTA group than in the NA group. Moreover, the RT for negative words was longer than for neutral words in the HTA group. The bars indicate standard deviations from the mean.

#### P300 data

Figure 2 presents ERP waveforms for negative emotional conditions in both the HTA and NA groups. A Group (HTA and NA)×Word type (negative, positive and neutral) ×Electrode site (C3, Cz, C4, P3, Pz, P4, O1, Oz and O2) ANOVA was conducted for P300 amplitude and latency. The main effect of electrode site was significant for P300 amplitude (F(1, 51) =22.34, *p*<0.001). However, the main effects of word type and group were not significant (*p* > 0.05). The interaction between electrode site and group was significant (F(2, 60)=4.31, *p*=0.023), and simple-effect tests found that P300 amplitudes induced in the P3 site were higher in the HTA group than in the NA group (F(1, 35)=10.87, *p*=0.002).

**Figure 2:** **Grand-average ERP waveforms evoked by negative words in the EST in both the HTA and NA groups.** Simple-effect tests indicated longer P300 latencies in the HTA group than in the NA group.

The main effect of electrode site was significant for P300 latency (F(1, 52) = 8.31, *p*= 0.002). The interaction between word type and group was significant (F(1, 47)=3.88, *p*=0.044), and simple-effect tests found that P300 latencies induced by negative words were longer in the HTA group than in the NA group (F(1, 35)=6.43, *p*=0.016). However, there was no significant difference of the P300 latencies for positive (F(1, 35)=0.04, *p*=0.85) and neutral words (F(1, 35)=0.10, *p*=0.75) between the HTA and NA groups (Figure 3). The interactions of word type, electrode site and group were significant (F(2, 82)=7.14, *p*=0.001). A follow-up with between-group contrasts for each emotional condition revealed that P300 latencies for negative words at Pz and Oz sites were longer in the HTA group than in the NA group (Pz: t(35)=4.30, *p*=0.046; Oz: t(35)=10.89, *p*=0.002).

**Figure 3:** **Grand-average ERP waveforms evoked by positive and neutral words in the EST in both the HTA and NA groups.** There was no significant difference of the P300 latencies for positive and neutral words between the HTA and NA groups.

### Experiment 2

#### EEG biofeedback data

There were no statistically significant differences between EEG BF and sham-BF groups for gender, age, TAI’s score,RT,P300 amplitude and latency in the EST (*p* >0.05). After all of the training sessions, TAI’s scores were significantly decreased by 10.28±4.33 in the EEG BF group (t(11)=4.23, *p*=0.03) while the sham-BF group rendered a decrease, though not significant, of 5.12±3.05. Furthermore, TAI's scores were significantly lower in the EEG BF group than in the sham-BF group after the intervention (t(21)=−3.17, *p*=0.04). The results of the intervention on the EST are shown in Figure 4. A Word type (negative, positive and neutral)×Group (EEG BF and Sham-BF)×Time (pre- and post-intervention) mixed-design ANOVA revealed a significant Time main effect for RTs (F(1, 35)=5.56, *p*=0.016). The interaction between word type and group was significant (F(2, 70)=3.45, *p*=0.037). The analysis of the alpha amplitudes' baseline value indicated that alpha amplitudes were significant enhanced post-training compared to pre-training in the EEG BF group(t(11)=5.36, *p*=0.01), while no significant changes were found in the sham-BF group.

**Figure 4:** **Changes in attentional bias to negative words pre- and post-intervention of EEG BF and sham-BF.** In contrast to the sham-BF group, a significant reduction in RT for negative words during the EST was evidenced in the EEG BF group. The bars indicate standard deviations from the mean.

The ANOVA analysis for P300 amplitudes in the pre- and post-intervention revealed no significant differences within the EEG BF and sham-BF groups (*p* > 0.05).

The mixed-design ANOVA for P300 latencies in the EST disclosed a significant Word type×Time×Group interaction effect (F(1, 47)=3.68, *p*=0.024). Simple-effect tests found that P300 latencies evoked by negative words were shortened after the intervention in the EEG BF group (F(1, 35)=6.24,*p*=0.018), whereas there were no differences in P300 latencies toward positive and neutral words between pre- and post-training. The Word type×Electrode site×Group interaction effect was significant (F(2, 82)=7.14, *p*=0.001). At the single electrode level, the EEG BF group displayed a significant reduction in the P300 latencies at Pz (t(11)=5.30, *p*=0.013) and Oz (t(11)=4.36, *p*=0.021). No significant changes were detected in the sham-BF group (Figure 5).

**Figure 5:** **Grand-average P300 waveforms (Pz) evoked by negative words in the EST pre- and post-training of EEG BF and sham-BF.** After the intervention, there was a significant decrease in the P300 latency at Pz to negative words in the EEG BF group, while no significant changes were present in the sham-BF group.

## Discussion

Consistent with previous studies [5,26,27], we found that attention performance can be modified by negative words in HTA individuals in the emotional Stroop task. Singhal et al. found that the P300 amplitude was larger for emotional pictures (fear and sadness) than for neutral pictures in anxious adolescents during the emotional oddball paradigm [28]. The current study showed that the P300 latency induced by negative words was longer in the HTA group than in the NA group. This P300 delay can be interpreted as reflecting the sustained negative-related emotion processing in HTA individuals.

This study examined the efficacy of EEG BF on attentional bias in HTA. Anxious individuals were trained to increase alpha amplitudes. The improvement of attentional bias was confirmed, as the RT toward negative words of the EST was significantly less in the EEG BF group than in the sham-BF group. A significant reduction in the TAI’s scores was also observed after the EEG BF group was given alpha training. The present study demonstrated that the improvement in anxiety observed in the EEG BF group were not merely due to general relaxation training, as these benefits were not observed in the sham-BF group. The sham-BF group experienced the same relaxation strategy as the EEG BF group but was provided with a non-feedback reward. Recent research has shown promising results in anxious children and adults by using attentional bias modification training [29-31]. To explore the optimising procedure, future studies are expected to compare different interventions on attentional bias.

The present findings support alpha amplitude as a promising EEG BF parameter that is worth exploring and investigating further. Alpha may reflect the resonance frequency of such a feedback loop for the state of an optimal cognitive performance. Most individuals reported evoking relaxation as the best strategy to increase alpha. Recent studies indicated that long-range upper alpha band synchrony is well suited to serve attention in cognitive function [32]. These findings could also explain varieties of training successes across studies. Personality factors, the alpha distribution or the impact of cognition could be individual factors predicting or influencing the success of EEG BF. The different findings in current and prior studies using EEG BF could arise from the many differences among these studies, including differences in methodology (alpha vs. SMR, beta training) and/or sample characteristics (anxiety vs. healthy) [9,13,14,33]. Alpha training alone cannot fully explain the effects of EEG biofeedback. Therefore, using different frequency bands for training would be desirable for future studies.

This study provides some evidence of the intervention effect of EEG biofeedback. Moreover, the study also generates some insights into the mechanism by which EEG biofeedback improves attentional bias toward negative stimuli. The present study suggests that improved control of attention on negative stimuli contributes to the observed emotional benefits of HTA as a direct effect of EEG biofeedback, which is possibly achieved through the effects on the reduction of P300 latency. In addition, P300 latencies of the EEG BF group were significantly shorter post-training than pre-training, which was not observed in the sham-BF group, supporting a relationship between P300 latency and attention performance. Previous studies demonstrated that P300 evoked by target stimuli was generated mainly at the posterior cingulate cortex and could reflect the high cognitive activation and attention [23]. Although the statistical analysis did not show a main effect of EEG biofeedback on the P300 latency in the EST, alpha training led to the reduction of P300 latency to negative stimuli at parietal and occipital lobes in HTA individuals. The modulation process may be involved in cognitive information communication among these activated regions from alpha sources (occipital lobe) to P300 generators (posterior cingulate cortex). This finding indicates that alpha activity appears earlier than P300 for attention processing. Further studies are needed to elucidate the underlying mechanisms of EEG biofeedback on these effects.

A small sample size in this study might limit the generalization of practical application and necessitates replication of these findings. Negative stimuli rather than threat stimuli were employed for HTA individuals, which could attenuate outcomes and limit generalisability to other affective stimuli. While alpha training is somewhat akin to SMR or beta training paradigms, the use of other training paradigms may raise questions whether these findings could be explained by an artifact related to specific differences between different frequency band training. While these questions cannot be resolved by the present data, it should be noted that there are no strong theoretical grounds for predicting that specific differences in different paradigms would explain the observed reduction in clinical anxiety or the increased attention bias to negative stimuli. Further studies with larger sample sizes are required to clarify these alternative explanations.

## Conclusions

This study demonstrated that the P300 latency was prolonged to negative words in HTA individuals, which is associated with attentional bias. EEG biofeedback can improve the anxious state and negative emotional attentional bias in HTA individuals. The mechanism of EEG biofeedback intervention may be related to the normalization of P300 latency. Our findings have shown the effectiveness of EEG biofeedback training on the high trait anxiety group.

## Abbreviations

HTA: High trait anxiety; NA: Nonanxious; EEG: Electroencephalogram; ERP: Event-related potential; S-TAI: State-trait anxiety inventory; EST: Emotional stroop task; BF: Biofeedback; RT: Reaction time.

## Competing interests

The authors declare that they have no competing interests.

## Authors’ contributions

WS contributed to the EEG biofeedback training, ERP recordings, data analysis and wrote the manuscript with ZY and CSJ. LGP and SP participated in the design and analysis of the data. WTH acquired the funding and contributed to the study design. All authors read and approved the final manuscript.
